# Brains, innovations, tools and cultural transmission in birds, non-human primates, and fossil hominins

**DOI:** 10.3389/fnhum.2013.00245

**Published:** 2013-06-06

**Authors:** Louis Lefebvre

**Affiliations:** Department of Biology, McGill UniversityMontréal, QC, Canada

**Keywords:** brain, innovation, tool, cultural transmission, bird, non-human primate, hominin

## Abstract

Recent work on birds and non-human primates has shown that taxonomic differences in field measures of innovation, tool use and social learning are associated with size of the mammalian cortex and avian mesopallium and nidopallium, as well as ecological traits like colonization success. Here, I review this literature and suggest that many of its findings are relevant to hominin intelligence. In particular, our large brains and increased intelligence may be partly independent of our ape phylogeny and the result of convergent processes similar to those that have molded avian and platyrrhine intelligence. Tool use, innovativeness and cultural transmission might be linked over our past and in our brains as operations of domain-general intelligence. Finally, colonization of new areas may have accompanied increases in both brain size and innovativeness in hominins as they have in other mammals and in birds, potentially accelerating hominin evolution via behavioral drive.

Neuroscientists and paleoanthropologists use very different approaches to study the relationship between intelligence and the brain. While neuroscientists study variance between contemporary individuals and species, drawing on techniques like brain imaging, intelligence tests and comparative analyses, paleoanthropologists focus mostly on variation over time and space in fossils and artifacts, in particular tools. This emphasis gives paleoanthropologists a unique insight into three key features of human intelligence: *innovation*, the first appearance of a novel technique or behavior, *tool* use and manufacture, and *cultural transmission*, the diffusion of innovations over space and time.

Studies of tools, innovations and cultural transmission in relation to avian and non-human primate brains have become more numerous in recent years. In this chapter, I review these studies and argue they are relevant to the neuroscience of hominin^1^ evolution. More specifically, the studies suggest that (1) large brains and increased intelligence in hominins may be partly independent of our ape phylogeny: convergence with avian and platyrrhine cognition, not just ape cognition, may be relevant to understanding our own; (2) tool use, innovativeness and cultural transmission might be linked over our past and (3) in our brains; (4) colonization of new areas may have accompanied increases in both brain size and innovativeness in hominins as they have in other mammals and in birds, potentially accelerating hominin evolution via behavioral drive.

## Variation in innovation rate is highly skewed toward a few phylogenetically independent taxa

If, in archeology, cultures carry the name of the first site where they were discovered, Swaythling and Koshima should feature prominently in the terminology of non-human cultures. In 1921, blue tits in Swaythling, a town near Southampton, were first seen to open milk bottles on doorsteps and drink the cream accumulating at the top. By 1949, the behavior had been noted in hundreds of localities throughout England, Wales, and Ireland (Fisher and Hinde, 1949). In the 1950's, a young female macaque on the Japanese island of Koshima innovated two food-washing techniques (potato washing in 1953 and wheat placer mining in 1956) that were later seen in several members of her troop (Kawai, 1965).

For decades, the main preoccupation of researchers was whether or not the “Swaythling bottle opening culture” and the “Koshima food washing culture” were truly cultures, i.e., whether social learning was behind the increase in the behaviors over time. Critical discussions (Hinde and Fisher, 1951, 1972; Galef, 1992; Ingram, 2001; de Waal, 2003), experiments on captive animals (Sherry and Galef, 1984, 1990; Kothbauer-Hellmann, 1990; Visalberghi and Fragaszy, 1990; Aplin et al., 2013) and statistical models of diffusion over space and time (Lefebvre, 1995a,b) were all concerned with transmission, but no one really asked why the innovations occurred in tits and macaques in the first place. When, decades later, innovation rates were calculated in birds and primates, tits and macaques were among the top genera: the genus *Macaca* is surpassed only by *Pan, Pongo*, and *Cebus* in Simon Reader's primate database (Reader and Laland, 2002; Reader et al., 2011), while the tit genus (formerly *Parus*, now split into *Parus, Poecile*, and *Cyanistes*) is eighth out of 362 genera with at least one innovation in the avian database collated by my lab (see supplement in Overington et al., 2009, 2011).

Overall, the primate and avian data sets show two clear and similar trends: first, some species have much higher innovation rates than others, and second, high innovation species are found in distant parts of the phylogenetic tree of their class or order. In primates, 60% of all innovations occur in a single species, the common chimpanzee. When the innovations of orang-utans and gorillas are added to the chimpanzee total (bonobos do not appear in the Reader database because they are so difficult to study in the field), the proportion of innovations that occur in great apes goes up to 75%. The genera *Cebus, Papio*, and *Macaca* together contribute another 20%. If baboons and macaques are not very distant in terms of molecular phylogeny (tribe *Papionini*), the group they belong to, the *Cercopithecinae*, is clearly very distant from the lineages that led respectively to *Cebus* and the great apes (see Figure 1B in Reader et al., 2011).

Simple counts of innovation frequency might not be the best way to compare taxa because they are probably biased by many factors. Species that are more populous than others or on which more research is conducted might yield more cases of innovative behavior. Up to now, thirteen such biases (often correlated with each other) have been shown to occur in studies of avian and primate innovation, but they are easily corrected by including the most important ones as confounding variables in multivariate analyses (Lefebvre et al., 2001; Lefebvre, 2011). When the main bias, research effort, is taken into account, the same primate genera as before yield the highest residual innovation rates, except for *Macaca*. Chimpanzees and orang-utans show standardized residuals that are clear outliers, respectively, 4 and 3.5 standard deviations above the primate average. High innovativeness thus seems to have evolved three or four times independently in primates: in the great ape lineage, the capuchin lineage and the baboon and macaque lineage (see Figure 1B in Reader et al., 2011). The capuchin lineage has been evolving separately from that of *Hominidae* and *Papionini* for more than 40 million years.

In birds, the distribution of innovations is also skewed toward some taxa. The families *Corvidae, Accipitridae* and *Laridae* rank at the top with over 200 innovations each, but none dominates the way great apes do in primates (Lefebvre et al., 1997; Overington et al., 2009). In birds, the ten genera with the highest innovation frequencies make up only 30% of the more than 2300 cases recorded. The taxonomic distribution of innovation rate is a bit more skewed at higher levels, but again less so than in primates. At four standard deviations above the avian mean, the *Corvoidea* superfamily (crows, shrikes, magpies, drongos, jays) is the clear outlier in birds when innovation rate is expressed as a residual of research effort, but even then, its innovation frequency represents only 15% of the avian total. Within this parvorder, the genus *Corvus* (ravens and crows) is an outlier at over eight standard deviations above the avian mean, by far the highest of all genera. Other avian clades with large residual innovation rates are raptors, woodpeckers, hornbills, gulls, kingfishers, roadrunners, and herons. Estimates of phylogenetic distances between these groups have changed drastically over the past 25 years, but innovation trends have proven robust (Overington et al., 2009) to major revisions, e.g., from the Sibley and Ahlquist (1990) phylogeny to the one published by Hackett et al. (2008).

In birds, variation in innovativeness has only been studied at the species level and higher, but in primates, Reader and Laland (2001) have also examined potential differences between males and females, as well as differences between juveniles and adults and high- vs. low-ranking individuals. Imo, the most famous primate innovator, was a high-ranking juvenile female when she invented potato and wheat washing, but trends in primates as a whole and in chimpanzees in particular do not confirm the picture seen at Koshima. In primates in general and in chimps in particular, males innovate significantly more than females when we take into account the sex ratio of the populations, which is often female biased; when sex ratio is not included in the analysis, males and females innovate at rates that are not significantly different. Across all primates, adults innovate more often than juveniles; in chimps, however, there is no significant difference between the two age classes. In chimps, as well as in primates in general, low ranking individuals innovate more frequently than mid- or high-ranking individuals.

The data on non-humans thus suggest two possibilities behind the high innovation rate of *Homo*: a trait that is phylogenetically shared with our hominid cousins, but also a trait that might have been influenced by convergent, independent evolution under pressures similar to those that favored innovativeness in *Cebidae, Corvidae*, and other taxa.

## Innovation, tool use and social learning: co-evolved cognitive modules or general intelligence?

In archeology, the study of tools, innovations and cultural transmission often go together. Recent analyses (Lycett and von Cramon-Taubadel, 2008; Lycett and Norton, 2010) on geographic distributions of lithic technologies, for example, focus on different modes of tool making, dates and loci of innovations (e.g., first appearance in Africa) and models of cultural transmission from the African areas of innovation to the farthest points of diffusion east of the Movius line. The study of tool use, innovation and cultural transmission also go together in quantitative counts of cognition in birds and primates. Using the same method to gather case studies on tool use and social learning (the mechanism that allows cultural transmission) as they did on innovations, Reader and Laland (2002) found significant positive correlations between the taxonomic distributions of the three measures. As with innovations, the great majority of tool use cases are found in *Pan, Pongo*, and *Cebus*; the three genera together make up 96% of recorded cases. The trends are maintained after correction for research effort: *Pan, Pongo*, and *Cebus* have corrected tool use rates that are 2–5 standard deviations above the average primate line.

This strong skew in the taxonomic distribution of primate tool use is also reflected in the avian database. Seventy-two percent of cases in the feeding domain (Lefebvre et al., 2002) and 87.5% of cases in all tool use domains (Bentley-Condit and Smith, 2010) are found in songbirds, the suborder *Passeri*. The genus *Corvus* once again stands out: fifteen species in this genus feature at least one tool use technique, with the New Caledonian species *Corvus moneduloides* showing the most sophisticated forms of use, manufacture and invention, as well as a causal understanding of tools, meta-tools and proto-tools (Taylor et al., 2009).

Quantitative counts of social learning in primates follow the same trends as do innovations and tool use. Again, chimpanzees and orang-utans clearly dominate, making up 68% of cases between the two of them and reaching 3–4 standard deviations above the mean primate line when corrected for research effort. *Cebus* scores a bit lower on this measure than it does on innovation and tool use, while *Macaca* (especially *M. fuscata*, the Japanese macaque on which extensive social learning research has been done) scores slightly higher with over 10% of primate cases. In birds, there are surprisingly few recorded cases of social learning of foraging behavior in the field. In primates, reports of innovation and social learning are about equally frequent, but in birds, there are less than 100 social learning reports (vocalizations excluded from this measure) for over 2300 innovation reports (Lefebvre and Bouchard, 2003); most are concentrated in the songbird suborder *Passeri*.

Taxonomic counts of tool use and innovation are positively correlated in both birds (Lefebvre et al., 2002) and primates (Reader and Laland, 2002; Lefebvre et al., 2004). This could be an artifact of a common bias in the collection method for the measures, as both are based on systematic surveys of the anecdotal literature. However, the fact that the measures also correlate with experimental results from captive animals argues against this possibility. In birds, differences in reversal learning errors between species from seven families correlate with both innovation rate and size of the mesopallium (Timmermans et al., 2000), while differences in problem-solving between five species of West Indian birds correlate with differences in innovation frequency (Webster and Lefebvre, 2001; Lefebvre and Bolhuis, 2003). In primates, differences in innovation rate also correlate with differences in reversal learning in six species [(Lefebvre et al., 2004); based on Riddell and Corl (1977) and Reader and Laland (2002)], and in nine types of cognitive tasks in 24 genera (Deaner et al., 2006; Reader et al., 2011).

Reader et al. (2011) have explored the idea of general intelligence with a principal components analysis that included five measures of cognition, adding Byrne and Whiten's (1987) tactical deception and Parker and Gibson's (1979; Gibson, 1986) extractive foraging to innovation, tool use and social learning, as well as three lifestyle or socio-ecological measures (diet breadth, percent frugivory, and group size). All five cognitive variables clustered together on the first PC, while the three lifestyle measures clustered on a second, independent, PC. This suggests that some form of general intelligence (abbreviated as *g* in the literature, e.g., Colom et al., 2006) might underlie the evolution of the different cognitive measures. Interestingly, the idea that animal intelligence includes distinct social and non-social domains was not supported in Reader et al.'s analysis: instead of a split between social variables (social learning, tactical deception, group size) and non-social ones (tool use, extractive foraging, and diet), the PCA revealed independent lifestyle and cognitive factors, whether social or not. Deaner et al. (2006) came to the same conclusion as Reader et al. (2011): a common general intelligence factor seems to underlie the co-variation in performance over the nine types of cognitive tasks they analyzed in 24 primate genera (see, however, Amici et al., 2012).

The implication for hominins are that cognitive traits such as innovativeness, tool use, social learning, tactical deception and reversal learning might all have evolved together. For many years, the dominant view in evolutionary psychology has been that cognition is best understood as a mental tool kit that includes several independent modules, each specialized for a particular purpose (Samuels, 2000; Shettleworth, 2010). While some cognitive features in non-humans seem to be modular (e.g., specialized, domain-specific and based on a dedicated neural substrate, such as filial imprinting, song, and spatial memory), other cognitive abilities could be better understood as domain-general processes. The positive correlations across species suggest that there are few trade-offs and that a species that ranks high on one cognitive measure can rank high on others. Chiappe and MacDonald (2005) have argued that selection for modular specializations depends on repeated encounters with situations that select for them (e.g., repeated winters killing birds that do not store food efficiently). By definition, this cannot be the case for innovation, which constantly deals with new problems rather than repetitions of the same one. Resource defense and game theory further predict that the spatial and temporal unpredictability of food should drive social and ecological intelligence in similar directions (Overington et al., 2008), which argues for concerted selection on multiple cognitive domains rather than strict modular specialization. If we add to this evidence from brain imaging (Colom et al., 2006; Barbey et al., 2012), genetics and intelligence test research in contemporary humans (Plomin and Spinath, 2002) and non-humans (Galsworthy et al., 2002), it is plausible that changes in *g* might lie behind many cognitive innovations found in our hominin past. Recent papers by Deaner et al. (2006), Byrne and Bates (2007) and van Schaik et al. (2012) have underlined this new interest in general vs. modular processes for the evolution of intelligence. It should be noted here that acknowledging the existence of *g* in no way implies that it accounts for all (or even most) of the variance in performance over different tasks across clades. In humans and other mammals, the proportion of variance explained by the first PC on a battery of cognitive tests is usually around 40% (Chabris, 2007), leaving a majority of the variance unexplained or associated with task- or domain-specific effects.

## Big brained birds and primates have higher rates of innovation, tool use, and social learning

Several neural measures are used in comparative studies of non-human cognition. The measures vary in the neuroanatomical level they focus on and the extent to which body size allometry is controlled for. In birds, innovation and tool use rates are positively correlated with allometrically corrected size of the whole brain, of the telencephalon and of the mesopallium and nidopallium, two areas that show convergent evolution with association areas of the mammalian cortex (Timmermans et al., 2000; Mehlhorn et al., 2010; Güntürkün, 2012). They are not correlated with absolute size of the brain, due to the presence of very large-bodied groups with poor cognitive skills such as ostriches, emus, bustards, and turkeys. Neither the anatomical level used (whole brain, telencephalon, or mesopallium and nidopallium) nor the method used to correct for body size (residuals, EQ or executive brain ratio) have an effect on the magnitude of the relationship between innovation rate and neural substrate (Lefebvre and Sol, 2008). In primates, innovation and tool use also co-vary, as well as correlate positively with absolute and allometrically corrected size of the isocortex. Taxonomic differences in social learning also correlate with isocortex size, as well as with rates of tool use and innovation (Reader and Laland, 2002).

One caveat is that these correlations, despite being highly significant, do not account for a large proportion of variance. In birds, residual brain size at the family level explains only 13.4% of the variance in diversity of technical innovations, the best measure of innovativeness in Overington et al. (2009) re-analysis of the avian database. In primates, the magnitude of the relationship between brain size and cognitive measures accounts for 13–18% of the variance when phylogenetic relatedness between taxa is taken out of the analysis (Reader and Laland, 2002). What this implies is that enlarged brains might be a necessary, but not a sufficient, factor in explaining innovativeness, tool use and social learning, whether this is in non-humans or in hominins. Other factors, be they environmental (e.g., spatially and temporally unpredictable resources) or behavioral (e.g., boldness, low neophobia) need to be considered.

In non-human primates, up to 26 different measures have been used to document lifestyle, cognitive, life history and evolutionary predictors of encephalization [reviewed in Lefebvre (2012)]. These range from log absolute mass of the whole brain, to the ratio of non-visual cortex volume divided by volume of the rest of the brain minus the cerebellum, to residuals of isocortex volume regressed against brainstem volume. Eighteen of the 26 measures use some measure of isocortex volume, removing or not the visual areas and adding or not the volume of the striatum. Structures used in allometric corrections of isocortex volume include the whole brain, the medulla, the brainstem (mesencephalon plus medulla oblongata), and the brain minus the isocortex (usually termed “rest of brain”).

In hominins, fossil data are almost always limited to estimates of endocranial volume, often inferred from incomplete crania (note that shape can also be analysed in some cases, e.g., Bruner, 2004; Gordon et al., 2004). We thus cannot do largescale analyses on hominins using the most popular structure for non-human primates, the isocortex, nor correct for allometry with intra-brain measures like the brainstem or the “rest of brain.” Largescale tests on hominins can only be done on whole brain size and allometric corrections done with body size, which can be selected naturally or sexually independently of brain size and vary more than the brain as a consequence of nutrition and disease. These limitations must be kept in mind when comparing variation in hominin brain size with that of non-human primates.

Henneberg and colleagues (Mathers and Henneberg, 1996; Henneberg, 1998; de Miguel and Henneberg, 1999, 2001; Henneberg and de Miguel, 2004) have collated the available data for brain and body size in hominins from 3.2 million to 10,000 years BP. Absolute values from their database are plotted in Figures 1A,B, excluding robust species *Paranthropus, Australopithecus boisei*, and *A*. *robustus*. Brain size is plotted as absolute volume, to emphasize the constant increase over time, while body size is plotted as log transformed kg, to emphasize the variation, both within and between time periods that is much larger than that of brain size. Some of the values (blue triangles) on the body size graph are so large that they represent outliers, possibly very large males in periods of high sexual dimorphism. The absence of similar outliers in the brain size graph is typical of dimorphism trends in non-human primates, where large sex differences in body size are often accompanied by small differences in brain size.

**Figure 1:** **Hominin brain and body size as a function of time from 3.2 million to 10,000 years BP.** Data from Henneberg and colleagues, excluding robust species and data points for which species identity is uncertain. **(A)** Absolute brain size in cc. **(B)** Log transformed body size in kg; triangles in **(B)** represent very large individuals.

Henneberg and de Miguel (2004; see their Figure 1) point out the continuous nature of the parallel trends in brain and body size over time. If we were working with birds or non-human primates, however, we would examine actual allometrically corrected encephalization measures, using either residuals of log brain size regressed against log body size or ratios, which can be calculated as simple brain mass divided by body mass or as EQ, the ratio of observed brain mass divided by the mass expected for the average member of body size × in a given taxonomic group. Brain and body estimates in such cases are normally taken from the same individuals; alternatively, brain mass is measured from fresh tissue or endocrania, and body mass taken from a standard source of species-typical mass, for example Dunning (2008) for birds. For hominins, the problem is that fossils used for brain and body size estimates are rarely from the same individual. We thus cannot simply match an individual brain size data point with its matching body size in the Henneberg database.

One solution is to use the gaps in the fossil record and the divisions in hominin clades to calculate a series of average brain and body masses for particular time periods. Table 1 presents one way of dividing the fossil record into time periods. It separates the clades recognized in Henneberg's database (*Australopithecus afarensis, A. africanus, Homo habilis, H. erectus*, archaic *Homo sapiens, Neanderthal*, and modern *H. sapiens*), eliminating cases where species identification is uncertain [e.g., entries 114–123 in de Miguel and Henneberg (1999)]. Given the long history of *H. erectus* and the large amount of body size variation seen in this clade, the table separates this species into four time periods.

**Table 1:** **Brain and body size averaged for time periods and clades (data based on Henneberg and colleagues)**.

**Clade**	**Time span (*k* years BP)**	**Mean time (*k* years BP)**	**Mean br (cc)**	**Mean body (kg)**
af	3200–3246	3223	425.83	43.13
aa	2585–2622	2603	477.24	43.20
hh	1803–1855	1829	635.98	51.44
he	1612–1682	1647	882.11	49.50
he	1137–1250	1193	890.37	60.00
he	877–884	881	883.32	68.30
ahs	612–650	631	1224.66	52.80
he	323–400	362	1066.53	51.66
n	47–51	49	1496.50	60.00
hs	38–40	39	1471.22	66.25

Abbreviations: af, Australopithecus afarensis; aa, Australopithecus africanus; hh, Homo habilis; he, Homo erectus; ahs, archaic Homo sapiens; n, Neanderthal; hs, Homo sapiens.

Figures 2, 3 illustrate the changes over time in the averaged data. Figure 2 shows averaged absolute brain and body size over the clades and periods. The validity of the divisions in Table 1 is supported by the small standard errors of the mean for time periods and brain size; in line with the large amount of body size variation obvious in Figure 1B, SEM's in Figure 2B are quite large on the y-axis. Figure 3 shows averaged allometrically corrected brain size according to four methods: brain/body ratio, EQ according to Jerison's (1973) formula, EQ according to Martin's (1981) formula and residuals of log brain regressed against log body size. In the last case, a reference group is required to yield the regression line with respect to which a hominin data point is to be compared. Here, I use brain and body size for contemporary Catarhines (apes and Old World monkeys), the clade that hominins belong to, adding to this data set the hominin data point for a given period and repeating the regression for each time and/or clade division in Table 1.

**Figure 2:** **Changes over time in absolute brain and body size averaged for periods and clades. (A)** Absolute brain volume (in cc). **(B)** absolute body mass (in kg) over time. Data from Henneberg and colleagues; errors bars on the x and y axes represent SEM's. Abbreviations above each data point in **(A)** correspond to the ten clades in Table 1; data points in **(B)** as in **(A)**.

**Figure 3:** **Changes over time in allometrically corrected brain and body size averaged for periods and clades. (A)** Brain size corrected for body size according to Jerison's EQ. **(B)** Brain size corrected for body size according to Martin's EQ. **(C)** brain/body ratio. **(D)** Studentized residuals of log brain size regressed against log body size. Data points as in Figure 2.

The striking thing about Figures 2, 3 is that all methods yield the same qualitative trends: the periods of maximum increase in both absolute or allometrically corrected brain size are the same: from 1.83 to 1.65, 0.88 to 0.63, and 0.36 to 0.05 My BP. This suggests that different ways of calculating hominin encephalization produce similar results, at least for the temporal and taxonomic divisions used here. Other ways of splitting the hominin data might yield different results, but the exercise attempted here at least supports the idea that the method used to calculate hominin encephalization trends does not have a strong effect on conclusions. The exercise also suggests that absolute hominin brain size yields similar temporal trends to those obtained with allometric corrections.

Two of the cognitive measures known to correlate with encephalization in birds and non-human primates, innovation and tool use, can be compared to the temporal trends in hominin brain size. Stout (2011) has proposed an ordinal scale of complexity changes over time for hominin tool innovations. The measures of complexity are based on archeological data, on inferences concerning mental operations, as well as observations and brain imaging of skilled contemporary stone toolmakers (Stout and Cheminade, 2007, 2009, 2012; Stout et al., 2011). The scale, albeit ordinal on the y-axis, fits remarkably well with Henneberg's continuous data on absolute brain size changes over time (Figure 4).

**Figure 4:** **Ordinal tool complexity scale (red circles) from Stout (2011) plotted over absolute brain size (in cc) as a function of time from 3.2 million to 10,000 years BP.** Scale on right indicates ordinal increases in tool complexity. Abbreviations refer to categories in Stout (2011) Figure 2. UO, unifacial Oldowan; BO, bifacial Oldowan; KA, karari; CLCT, core LCT; FLCT, flake LCT; HC, hierarchical centripetal; CV, cleaver variants; RS, refined shaping; BL, blades; OP, other predetermined; LV, Levallois variants.

The overall message here is that hominin encephalization trends over time appear to be robust to the method used to estimate them, and that the relationship between tool use, innovations and brain size that shows convergent co-evolution in birds and non-human primates [see Figure 2 in Lefebvre et al. (2004)] might also apply to hominins.

## Colonization and behavioral drive

In the early 1980's, Wilson and colleagues (Wyles et al., 1983; Wilson, 1985) proposed that the combination of innovatiness, social learning and large brains might have an accelerating effect on the pace of evolution. The example they used was that of the Swaythling bottle opening culture mentioned in the first part of this article. Birds do not digest the carbohydrates in milk, only the lipids. However, if a mutation in digestive enzymes were to occur that gave its avian bearer the equivalent of mammalian lactase, this mutation would easily become fixed in bottle opening birds, but not in birds that do not face a situation where the mutation provides an advantage. Once the lactase equivalent mutation results in a survival and reproductive advantage for the bearer and its descendants, several consequences may follow. First, any other trait that facilitates the one first selected might also be selected. Secondly, the new lines of lactose-digesting bottle openers might start diverging from their ancestral population, if only by the increased advantage they derive from urban and suburban habitats. The implication is that both the rate of evolution of different traits and the rate of divergence of populations may increase as a result of what Wilson and colleagues call “behavioral drive.” Mayr's (1965) idea that behaviorally flexible species might succeed better than conservative ones at invading new habitats complements Wilson's ideas quite well and leads to the prediction that innovative clades should be better colonizers and show a greater species and subspecies diversity than less innovative ones. Sol and colleagues have shown, for birds introduced to New Zealand (Sol and Lefebvre, 2000) and in other areas of the world (Sol et al., 2002, 2005a) that colonization success can be predicted by brain size and by innovation rate in the country of origin. Several species from the genus *Corvus*, the most innovative avian genus, have a very high colonization success and are considered pests, e.g., *Corvus splendens* in Africa, Singapore and the Arabian peninsula, *C. macrorhynchos* in Japan, *C. corax* in the American southwest. Successful mammal colonizers also have larger brains than unsuccessful ones (Sol et al., 2008), as do amphibians and reptiles (Amiel et al., 2011), but not fish (Drake, 2007).

The genus *Homo*, which Wells and Stock (2007) call “the colonizing ape,” has succeeded in invading almost every habitat on the surface of the earth, from the coldest to the hottest, from the driest to the wettest. Templeton (2002, 2005) has analyzed evolutionary trees of human haplotypes and pinpointed three major historical events that led to gene flow out of Africa, dated at approximately 1.9 million, 650,000, and 130,000 years ago. How do these dates compare to the temporal trends in brain size plotted in Figures 1, 2, 3? Repeated “out-of-Africa” events are reasonably close in time to the peaks in brain size, allometrically corrected or not, that characterize the averaged data per clade and time period. Figure 5A shows the three major “out-of-Africa” emigration events identified by Templeton's (2002, 2005) analyses plotted against residual brain size. The coincidence of these emigration events with continuous changes in absolute brain size over time is more difficult to see (Figure 5B).

**Figure 5:** **Dates of major hominin emigration events out of Africa (arrows) according to Templeton's (2002, 2005) plotted against (A) studentized residuals of log brain size regressed against log body size averaged for the time periods and clades presented in Table 1. (B)** Continuous change of log absolute brain size as a function of time from 3.2 million to 10,000 years BP.

One important factor behind Wilson's interest in behavioral drive was the possibility that evolutionary rates might vary between clades. Wilson was one of the pioneers of molecular clocks (Wilson et al., 1987) and famously proposed the “Mitochondrial Eve” hypothesis (Cann et al., 1987) as well as the 4–5 million years divergence date between the chimpanzee and hominin lineages (Wilson and Sarich, 1969). One prediction of behavioral drive is that large-brained, innovative taxa should show accelerated rates of evolution. Recent molecular analyses (Curnoe et al., 2006) suggest that speciation times for hominoids (0.66 My) were much faster than those that characterize other primates (1.1 My), as well as mammals in general (2.2 My, Avise et al., 1998). Accelerated speciation times, combined with the increased potential for separation of populations due to greater colonization success, might also lead to a higher diversification rate. In birds, the number of species (Nicolakakis et al., 2003) and subspecies (Sol et al., 2005b) per clade correlates with innovation rate and brain size. It is difficult to ascertain the number of species and subspecies in the hominin clade, but estimates based on fossils range from 5 species to 23, with a median of 14 (Curnoe and Thorne, 2003). Probability estimates also vary greatly from 8 to 27 species (Bokma et al., 2012). The possibility that several species and subspecies of hominins may have evolved and gone extinct over a relatively short timeline, as well as within overlapping periods, would be a logical extension of the behavioral drive hypothesis.

## Conclusion

This article attempts to summarize convergent trends in innovation, tool use, cultural transmission, and brain size in birds and non-human primates, and then see if the trends are useful in thinking about hominin evolution. Phylogenetic influences on hominin evolution have been the focus of much work, based on important field and captive studies of great apes, in particular chimpanzees and orangutans. Recent work on innovation and tool use in corvids (Hunt and Gray, 2003) and capuchins (Fragaszy et al., 2004) should remind us, however, that we have much to learn from thinking about hominin intelligence in terms of convergent, multiple independent evolutionary events. To understand the intelligence of *Homo*, the most invasive and opportunistic primate genus, an invasive and opportunistic avian genus like *Corvus* might be as useful as the currently dwindling and geographically limited populations of our closest sister taxa *Pan, Gorilla*, and *Pongo*.

### Conflict of interest statement

The author declares that the research was conducted in the absence of any commercial or financial relationships that could be construed as a potential conflict of interest.

## Footnotes

^1^The term “hominin” describes current humans and their immediate ancestors, while the terms “hominoid” and “hominid” include respectively apes and great apes.
